# Genetic variation in NOD1/CARD4 and NOD2/CARD15 immune sensors and risk of osteoporosis

**DOI:** 10.1042/BSR20192313

**Published:** 2020-07-02

**Authors:** Ahu Soyocak, Merih Özgen, Didem Turgut Coşan, Hülyam Kurt, Fulya Doğaner, Onur Armağan, İrfan Değirmenci, Fezan Şahin Mutlu

**Affiliations:** 1 Department of Medical Biology, Faculty of Medicine, Istanbul Aydin University, Istanbul, Turkey; 2 Department of Physical Medicine and Rehabilitation, Faculty of Medicine, Eskisehir Osmangazi University, Eskisehir, Turkey; 3 Department of Medical Biology, Faculty of Medicine, Eskisehir Osmangazi University, Eskisehir, Turkey; 4 Department of Biotechnology and Molecular Biology, Faculty of Arts and Sciences, Aksaray University, Aksaray, Turkey; 5 Department of Medical Biology, Faculty of Medicine, Kutahya Health Sciences University, Kütahya, Turkey; 6 Department of Biostatistics and Medical Informatics, Faculty of Medicine, Eskisehir Osmangazi University, Eskisehir, Turkey

**Keywords:** NOD1/CARD4, NOD2/CARD15, Osteoporosis, Polymorphism

## Abstract

The present study was aimed to investigate the relationship between NOD1/CARD4 and NOD2/CARD15 gene polymorphisms and osteoporosis in the Turkish population. The first time we thought that the functional polymorphisms in NOD1/CARD4 and NOD2/CARD15 genes might have triggered the development of osteoporosis. The objective of our study was to determine the relationship between NOD1/CARD4 and NOD2/CARD15 SNPs and osteoporosis. The NOD1/CARD4 (rs5743336) and NOD2/CARD15 (rs2066847) SNPs were analyzed by PCR restriction fragment length polymorphism (PCR-RFLP) in 94 healthy controls and 164 subjects with osteoporosis. PCR products were digested with restriction enzymes AvaI for NOD1/CARD4 and ApaI for NOD2/CARD15. We found that NOD1/CARD4 genotype distribution of AA, GA and GG were 15, 44 and 41% for patients and 17, 46 and 37% for controls, respectively. NOD2/CARD15 mutation was found only in three patients (1.8%) as heterozygote. The results did not show any statistical difference between NOD1/CARD4 and NOD2/CARD15 genotype distribution of patients and healthy groups (χ^2^ = 1.740, *P*=0.187; χ^2^ = 1.311, *P*=0.519). However, the most frequent AG genotype (46%) of NOD1/CARD4 was observed in healthy controls, GG genotype (44%) of NOD1/CARD4 was observed as the most frequent in osteoporotic patients. NOD2/CARD15 WT/WT genotype, the most frequent genotype, was observed in both groups. Statistical analysis revealed that NOD1/CARD4 and NOD2/CARD15 polymorphisms are not associated with osteoporosis. However, a definite judgement is difficult to be made due to restricted number of patients and small size of control group. Further research is sorely warranted in this direction.

## Introduction

Osteoporosis is a relevant age-related pathological disorder characterized by low bone mass, deterioration in the structure of the bone and increased bone fragility, that is chronic progressive disease, and negatively affects the quality of life [1]. This disease is mainly common in the elderly population, and an important public health issue that reduces the patient functioning and quality of life. An improved understanding of the risk factors for osteoporosis is important for the diagnosis, maintenance and treatment of this significant disease [2,3]. Several epidemiological and clinical studies have demonstrated the importance of genetics in osteoporosis pathogenesis [4–6]).

Genetic factors affect bone turnover and can result in the reduction in mass to ∼50–80% [4,6,7]. Gene polymorphisms may contribute to osteoporosis and impact bone mineral density (BMD) [7–12]. However, recently clinical and molecular study results emphasize that inflammation process also can effects on bone turnover in the osteoporosis [13–15]. Taken together, these findings suggested that the important link between inflammation and bone loss should be investigated genetically.

Nucleotide binding and oligomerization domain (NOD)-like receptors (NLRs) constitute a family of evolutionarily conserved cytosolic pattern-recognition molecules that bind exogenous and endogenous ligands [16,17]. NLRs are one of the major forms of innate immune sensors. These sensors’ respond against tissue damage, and activated sensors initiate tissue repair processes [18]. NOD1/CARD4 and NOD2/CARD15 are the members of NLR family and are located on chromosome 7p14-15 and 16q12, respectively. NOD1/CARD4 and NOD2/CARD15 play an important role in biological processes such as generating reactive oxygen species, apoptosis, autophagy and immune response [16,17]. NOD1/CARD4 is expressed by epithelial and myeloid-derived cells, while NOD2/CARD15 is primarily expressed in myeloid cells. However, NOD1/CARD4 also plays role in pathogen recognition, NOD2/CARD15 acts in the immune response against pathogenic organisms [16,17,19]. Besides this information, little is known about the role and mechanism of NOD1/CARD4 and NOD2/CARD15-induced innate immunity. However, genetic variants of NOD1/CARD4 and NOD2/CARD15 have been found to be associated with susceptibility to several inflammatory suggesting that these molecules are important in inflammation and immunity [16,18,20–28]. These genetic variants may influence the outcome of inflammation and osteoporosis. Furthermore, these proteins affect transcription factor, nuclear factor-κB (NF-κB) which plays an important role in age-related diseases [29]. NF-κB activation increases production of pro-inflammatory cytokine and its precursors and may affect the risk of developing infection, chronic inflammation, cancer and age-related diseases such as osteoporosis [29]. Recent studies suggest that there is a relationship between osteoporosis and periodontal disease, both diseases are characterized by bone loss [30–32]. Studies investigating the relationship between periodontal diseases and NOD1/NOD2 have shown that these proteins play a role in induction of innate immune responses and bone resorption [33–35].

Based on this relationship, it has been suggested that NOD variants may be associated with the risk of developing osteoporosis. We thought that the functional polymorphisms in NOD1/CARD4 and NOD2/CARD15 genes might have triggered the development of osteoporosis. The objective of our study was to determine the relationship between NOD1/CARD4 and NOD2/CARD15 SNPs and osteoporosis.

## Materials and methods

### Subjects

The study group included 258 postmenopausal females. The control group was composed of 94 healthy subjects (mean age: 50 ± 13) and the osteoporosis group was composed of 164 patients (mean age: 62 ± 8). Postmenopausal females who were admitted to the Osteoporosis Clinic of the Physical Medicine and Rehabilitation Department of Eskisehir Osmangazi University (Turkey) were informed of the study, and patients who opted for inclusion in the study were evaluated. The participants underwent dual-energy X-ray absorptiometry (DEXA) scanning using a Hologic QDR 4500 W system (Hologic, Inc., Bedford, U.S.A.) to assess BMD. Patients with a mean bone density below 2.5 SD were diagnosed with osteoporosis, as recommended by the World Health Organization (WHO). All participants underwent DEXA evaluations, and 164 postmenopausal females were diagnosed with osteoporosis based on this assessment. The study was approved by the Ethics Committee of the Medical Faculty of Eskisehir Osmangazi University (Turkey) (No. 80558721/310) and performed in accordance with the principles of the Declaration of Helsinki. Written informed consents were obtained from all subjects before the study.

### DNA isolation and genotyping

Genomic DNA isolation was performed using the salt-extraction method in 10 ml of peripheral blood that was collected in EDTA tubes for the analysis of NOD1/CARD4 (rs5743336) and NOD2/CARD15 (rs2066847) polymorphism. The association of NOD1/CARD4 and NOD2/CARD15 genes with osteoporosis was studied by PCR restriction fragment length polymorphism (PCR-RFLP). The PCR-RFLP of NOD1/CARD4 and NOD2/CARD15 polymorphisms amplified in a thermal cycler (Sacem Life Technologies, Peltier-based Thermal Cycler SCM 96G, Turkey) using 25 μl OneTaq® 2× Master Mix with Standard Buffer (New England Biolabs, Ipswich, MA, U.S.A.) according to manufacturer’s instructions. The reaction mixture contained 1 μl of genomic DNA, 0.5 μl of each primer (5 μM) (Alpha DNA, Montreal, Canada) (Table 1), 12.5 μl of Master Mix and 10.5 μl of nuclease-free water. The thermal cycle profile consisted of an initial denaturation step at 94°C for 30 s, followed by 35 cycles each consisting of three steps: denaturation for 30 s at 94°C, annealing for 60 s at 56,8°C for NOD1/CARD4 polymorphism and at 55,1°C for NOD2/CARD15, extension for 60 s at 68°C, and one elongation step at 68°C for 5 min. PCR products were digested for 1 h at 37°C by restriction enzymes, AvaI and ApaI (New England Biolabs, Beverly, MA, U.S.A.). Restriction enzyme digestion products were resolved by electrophoresis on 3% agarose gel. Gels were stained with RedSafe™ nucleic acid staining solution (Intron Biotechnology Inc., Seoul, Korea) and visualized using GeneGenius Gel Light Imaging System (Sygene, Cambridge, U.K.).

**Table 1:** PCR conditions and enzymes

SNPs	Primer sequences	PCR conditions	PCR products	Digestion products	Enzymes
**NOD1/CARD4 (rs5743336)**	F: 5′-TGAGACCATCTTCATCCTGG-3′ R: 5′-CTTCCCACTGAGCAGGTTG-3′	94°C, 30 s 94°C, 30 s 56,8°C, 60 s 68°C, 60 s 68°C, 5 min	379 bp	AA: 379 bp AG: 379 bp, 209 bp, 170 bp GG: 209 bp, 170 bp	Ava I 37°C 1 h
**NOD2/CARD15 (rs2066847)**	F: 5′-GGCAGAAGCCCTCCTGCAGGGCC-3′ R: 5′-CCTCAAAATTCTGCCATTCC-3′	94°C, 30 s 94°C, 30 s 55,1°C, 60 s 68°C, 60 s 68°C, 5 min	151 bp	WT/WT: 151 bp WT/insC: 151 bp, 130 bp, 21 bp insC/insC: 130 bp, 21 bp	Apa I 37°C 1 h

### Statistical analysis

The data were evaluated using SPSS Version 20 software (IBM Corp. Armonk, New York, U.S.A.). The continuous variables were not normally distributed based on the Shapiro–Wilk test for normality. The Mann–Whitney U test was implemented for mparison of the two groups. Medians (quartiles) were provided as descriptive statistics. The Pearson chi-square test was conducted for categorical variables. *n* and % values were provided. A *P*<0.05 was considered statistically significant.

## Results

In the present study, we found that NOD1/CARD4; genotype distribution of AA, AG and GG were 15, 41 and 44% for patients and 17, 46 and 37% for controls, respectively (Table 2). NOD2/CARD15 mutation was found only in three patients (1.8%) as heterozygote (Table 3). The results did not show any statistical difference between NOD1/CARD4 and NOD2/CARD15 genotype distribution of patients and healthy groups (c2 = 1.740, *P*=0.187; c2 = 1.311, *P*=0.519). Although the most frequent AG genotype (46%) of NOD1/CARD4 was observed in healthy controls, GG genotype (44%) of NOD1/CARD4 was observed as most frequent in osteoporotic patients. NOD2/CARD15 WT/WT genotype, the most frequent genotype, was observed in both the groups.

**Table 2:** Distribution of NOD1/CARD4 (rs5743336) genotypes

Groups	*n*	NOD1/CARD4 (rs5743336) genotypes					
		AA		AG		GG	
		*n*	%	*n*	%	*n*	%
Healthy controls	94	16	17	43	46	35	37
Osteoporotic patients	164	24	15	67	41	73	44
Total	258	40	32	110	87	108	81
Statistics	χ^2^=1.740, *P*=0.187						

**Table 3:** Distribution of NOD2/CARD15 (rs2066847) genotypes

Groups	*n*	NOD2/CARD15 (rs2066847) genotypes*			
		WT/WT		WT/insC	
		*n*	%	*n*	%
Healthy controls	94	94	36,9	0	0
Osteoporotic patients	164	161	98,2	3	1,8
Total	258	255	98,8	3	1,2
Statistic	χ^2^=1.311, *P*=0.519				

* The insC/insC genotype was not detected.

## Discussion

The NLRs, are intracellular innate immune molecules including NOD1/CARD4 and NOD2/CARD15 proteins that are essential for innate immune responses to bacterial infections and tissue injury. These cytosolic proteins respond to bacterial peptidoglycan intracellular fragments. These proteins also trigger gene transcription of NF-κB-dependent and mitogen-activated protein kinase (MAPK)-dependent [36]. Osteoporosis is a relevant age-related dysfunction, characterized by low bone density and increased bone fragility [1]. Recent times, the bone remodeling process-related study suggests that inflammation factors have a role in bone physiology and remodeling, according to this evidence inflammation importantly contributes to the pathogenesis of osteoporosis [37]. Different investigations indicate an increase in the risk of developing osteoporosis in various inflammatory conditions [38–41]. However, several diseases are related to osteoporosis [14] such as immunological dysfunctions, autoimmune and chronic inflammatory diseases [42], rheumatoid arthritis (RA) [43], hematological diseases [44], inflammatory bowel diseases [45,46] and periodontal disease [30,32,]. Although osteoporosis is not exactly qualified as an immunological disorder, recent studies have reported related molecular pathways between bone biology and biology of inflammation [14,47–49]. Pro-inflammatory cytokines play potential significant roles both in the normal bone remodeling process and in the pathogenesis of perimenopausal and late-life osteoporosis [14,50].

Osteoporosis, osteoarthritis and RA are most common musculoskeletal disorders. The major cellular integral of bone, osteoblasts, generate a bundle of immune molecules following bacterial challenge that could call leukocytes to infected areas and develop inflammation during bone diseases [51]. Marriott et al.’s study showed that murine osteoblasts expressed the novel intracellular pattern recognition receptors, NOD1/CARD4 and NOD2/CARD15. Levels of mRNA encoding Nod molecules and protein expression are greatly and disparately got higher from low basal levels following exposure to these different kinds of bacterial pathogens. As such, the presence of Nod proteins in osteoblasts could represent an important mechanism by which this cell type responds to intracellular bacterial pathogens of bone [51] However, RA is a specific case of the link between inflammation and osteoporosis. Pro-inflammatory cytokines and proteinases that are molecules involved in cartilage and bone destruction when released in joints and skeleton, there occurs bone loss in RA [52]. As a result, several studies suggest that NOD1/CARD4 and NOD2/CARD15 can have a significant role in the chronic and destructive inflammation of the joints in RA can regulate the innate immune response and may act a role in the continue of the inflammatory response in RA [53,54].

Genetic variations in NOD1/CARD4 and/or NOD2/CARD15 have previously been identified in many diseases such as inflammatory bowel disease [20,46], Crohn’s disease [22,24], sarcoidosis [23], non-Hodgkin lymphoma [21], cancer [16,26,27] and RA [55]. Plantinga et al. investigated the relation of the NOD1/CARD4 +32656 insertion/deletion polymorphism with RA [55]. The study results show that the NOD1/CARD4 +32656 polymorphism was not related with either susceptibility to, or clinical parameters of, inflammation or bone destruction in RA patients [55].

Osteoporosis, as well as other musculoskeletal and age-related disorders, has a strong genetic component and for this reason bone loss during senescence varies widely among different people [14]. The genetic mechanism underlying this disease process is largely unknown. Previous studies have investigated the NOD1/CARD4 and NOD2/CARD15 gene polymorphism in the many populations and several diseases. There are a few studies evaluating the association of these SNPs in Turkish population [25,27,28], while its relationship with osteoporosis has not been investigated in any population yet. In our study examined for the first time, relationship of the NOD1/CARD4 and NOD2/CARD15 polymorphism, which have a role in innate immune response with osteoporosis in Turkish women.

In our study, we also did not find a relationship possible with this polymorphism and osteoporosis. However, it has been observed for NOD1/CARD4 genes that AG genotype (46%) was the most abundant one in healthy controls whereas it was the GG genotype (44%) in osteoporotic patients. NOD2/CARD15 WT/WT genotype, the most frequent genotype, was observed in both groups.

## Conclusions

Our results suggest that the polymorphisms observed in the NOD1/CARD4 and NOD2/CARD15 genes are not genetic susceptibility factors for osteoporosis disease in Turkish women. However, this result may not be applicable to all populations when gene pools, lifestyles and gene–environment interactions in various populations are considered. Therefore, multicentered studies on different populations and in different gene regions in larger samples are required to establish the correlation between the NOD1/CARD4 and NOD2/CARD15 polymorphisms and osteoporosis. We believe that our results will contribute to the gene pool related to osteoporosis.

## Abbreviations

BMD: bone mineral density
CARD: caspase-recruitment domain
DEXA: dual-energy X-ray absorptiometry
NF-κB: nuclear factor-κB
NLR: nucleotide binding and oligomerization domain-like receptor
NOD: nucleotide binding and oligomerization domain
PCR-RFLP: PCR restriction fragment length polymorphism
RA: rheumatoid arthritis
SD: standard deviation
